RETRACTED

# LncRNA CCAT2 promotes the proliferation and metastasis of colorectal cancer through activation of the ERK and Wnt signaling pathways by regulating GNB2 expression

**DOI:** 10.1002/cam4.70169

**Published:** 2024-09-03

**Authors:** Jinhai Tian, Xu Cao, Zongying Jiang, Jia Wang, Wan Fan, Shaoting Zhang, Sien Zhao, Jianmin Sun

**Affiliations:** ^1^ School of Basic Medical Sciences Ningxia Medical University Yinchuan China; ^2^ Institute of Medical Sciences General Hospital of Ningxia Medical University Yinchuan China; ^3^ Department of Pathology General Hospital of Ningxia Medical University Yinchuan China; ^4^ Clinical Medical College of Ningxia Medical University Yinchuan China

**Keywords:** CCAT2, colorectal cancer, GNB2, metastasis, proliferation, signaling pathway

## Abstract

**Background:**

Colorectal cancer (CRC) is a prevalent and lethal tumor, with metastasis being the leading cause of mortality. Previous research has indicated that the long non‐coding RNA (lncRNA) CCAT2 is involved in the regulation of various tumor progression mechanisms. However, the precise role of CCAT2 in CRC proliferation and metastasis remains ambiguous. This study seeks to elucidate the mechanisms through which CCAT2 influences CRC.

**Methods:**

High‐throughput sequencing and RT‐qPCR were used to detect CCAT2 expression in CRC. Functional analyses including CCK8, colony formation, wound healing migration, transwell chamber, and Muse® Cell Analyzer assays were performed to study the effects of CCAT2 gene deletion on CRC cells. RNA‐pulldown and protein mass spectrometry were employed to identify the interaction between CCAT2 and GNB2 protein.

**Results:**

Increased CCAT2 expression was found in CRC, especially in metastatic CRC. Deletion of CCAT2 gene inhibited CRC cell proliferation, migration, and invasion while promoting apoptosis. The interaction between CCAT2 and GNB2 protein was shown to modulate GNB2 protein alterations and affect the ERK and Wnt signaling pathways, thereby promoting CRC proliferation and metastasis.

**Conclusion:**

CCAT2 plays a crucial role in CRC progression by modulating the ERK and Wnt signaling pathways through its interaction with GNB2. These findings highlight the importance of CCAT2 as a key regulatory element in the mechanisms underlying CRC proliferation and metastasis.

## 1 INTRODUCTION

Colorectal cancer (CRC) is a prevalent malignancy with a high global incidence and is a primary contributor to cancer‐related mortality.^1^ Despite advances in diagnosis and treatment, the high incidence of tumor recurrence and metastasis remains a major challenge in CRC management.^2^ Therefore, there is an urgent need to understand the molecular mechanisms underlying CRC progression and identify novel therapeutic targets. Long non‐coding RNAs (lncRNAs) have emerged as crucial regulators of gene expression and play significant roles in various biological processes, including cancer development and progression.^3^, ^4^, ^5^ The predominant mechanism of action attributed to lncRNAs in tumorigenesis thus far is the competitive endogenous RNA (ceRNA) mechanism, which impacts various aspects of tumor initiation and progression. This mechanism encompasses the modulation of oncogene expression, tumor biological processes, prognostic evaluation, and targeted therapeutic interventions.^6^ Additionally, certain lncRNAs have been implicated in conferring chemoresistance in CRC, such as the lncRNA CACClnc which facilitates chemoresistance through the regulation of RAD51 alternative splicing.^7^ Other lncRNAs regulate colorectal cancer progression through epigenetic modifications. Hypoxia‐induced lncRNA STEAP3‐AS1 activates the Wnt/β‐catenin signaling pathway and promotes CRC progression by preventing m6A‐mediated degradation of STEAP3 mRNA.^8^ The MYC‐activated lncRNA MNX1‐AS1 stabilizes YB1 and promotes colorectal cancer progression.^9^ Several long non‐coding RNAs (lncRNAs) have been identified to interact with key oncogenes or tumor suppressor genes, such as the P53 gene, thereby playing a role in tumorigenesis. The regulation of P53 by multiple lncRNAs has been shown to influence colorectal cancer carcinogenesis, tumor progression, and resistance to treatment.^10^ Our study has revealed that LncRNAs derived from Colon Cancer‐Associated Transcript 2 (CCAT2) are upregulated in CRC, with particularly pronounced upregulation in metastatic CRC. CCAT2 has been reported to be dysregulated in CRC and associated with poor prognosis.^11^, ^12^ However, the precise molecular mechanisms by which CCAT2 contributes to CRC proliferation and metastasis remain largely unknown. Guanine nucleotide‐binding protein subunit beta‐2 (GNB2) is a key signaling molecule involved in multiple cellular processes. Recent studies have implicated GNB2 in tumorigenesis and metastasis in several cancer types.^13^, ^14^ However, the role of GNB2 in CRC and its potential interaction with CCAT2 have not been thoroughly investigated.

RETRACTED

The objective of this study was to investigate the functional significance of the CCAT2‐GNB2 interaction in the progression and metastasis of CRC. Specifically, our research focused on elucidating the impact of CCAT2 binding to GNB2 on the activation of the ERK and Wnt signaling pathways, which play crucial roles in CRC pathogenesis. Our hypothesis posits that the CCAT2‐GNB2 interaction facilitates CRC proliferation and metastasis by modulating these signaling pathways. To test this hypothesis, a series of in vitro and in vivo experiments were conducted using CRC cell lines and animal models. Our findings provide novel insights into the molecular mechanisms underlying CRC progression and highlight the potential of targeting the CCAT2‐GNB2 interaction as a therapeutic strategy for CRC treatment.

In conclusion, the primary objective of this study was to investigate the functional importance of the CCAT2‐GNB2 interaction in CRC and its impact on tumor proliferation and metastasis through the regulation of the ERK and Wnt signaling pathways. A comprehensive understanding of the molecular pathways involved in CRC progression is essential for the advancement of targeted therapeutic approaches and the enhancement of patient outcomes in clinical settings.

## 2 MATERIALS AND METHODS

### 2.1 Tissue specimens

The research involved the collection of tumor tissues and corresponding adjacent non‐cancerous tissues from 117 patients diagnosed with colorectal cancer (CRC) at Ningxia Medical University General Hospital (Yinchuan, China), between June 2021 and March 2023. These patients met specific criteria, including no prior chemotherapy or radiotherapy treatment, absence of infectious diseases, or multiple malignancies. All patients were informed and provided written consent before inclusion. The experimental procedures were ethically approved by the Ethics Committee of Ningxia Medical University (Ethics Approval No: 2020‐626), and all procedures were conducted according to the principles outlined in the Helsinki Declaration.

### 2.2 Sequencing and data analysis

High‐throughput sequencing analysis of lncRNAs was conducted by Biomarker (Beijing, China), involving processes such as labeling, hybridization, scanning, normalization, and data analysis. The Ovation RNA‐Seq V2 kit was utilized for the comprehensive amplification of the transcriptome from RNA, with cDNA being generated through a single‐primer isothermal amplification method. Sequencing was carried out on the Illumina NovaSeq 6000 platform. Pathway analysis was performed using a combination of proprietary pathway analysis, R analysis, Gene Ontology (GO) enrichment analysis, and custom gene lists.

### 2.3 Cell culture

CRC cell lines, including HT29, HCT116, SW620 cells, and normal NCM460 cells, were obtained from the ATCC cell repository (Shanghai, China) and maintained in the laboratory of Ningxia Medical University General Hospital. McCoy 5A, L15, and RPMI‐1640 culture media (purchased from Gibco) were supplemented with 10% fetal bovine serum (Gibco) and 1% penicillin–streptomycin. Cells were cultured in a humidified incubator at 37°C with 5% CO_2_.

RETRACTED

### 2.4 RT‐qPCR

Total RNA from CRC cell lines or tissues was extracted using Trizol reagent (Invitrogen). cDNA synthesis was performed using the PrimeScriptTM RT reagent kit (Takara). RT‐qPCR was conducted using TB Green reagent (Takara) and the Roche 480 LightCycler PCR system. The following primer sequences were used: CCAT2 primers (F‐ AACCCCACAGTTCAGTTTCCT, R‐ TCTTGTTGGGACTTGCTGGTA); GNB2 primers (F‐ AGTGGGGATGTGATGTCCCT, R‐ GGTCTGTCGGCACATGGAAT).

### 2.5 Subcellular localization analysis

Fluorescence in situ hybridization (FISH) was utilized to examine the subcellular localization of CCAT2 by employing probes specifically designed and labeled with biotin to target the CCAT2 sequence. Following sample preparation and probe labeling, hybridization was carried out and the outcomes were assessed using fluorescence microscopy. The Cytoplasmic & Nuclear RNA Purification Kit (NORGENBIOTEK, Canada) was utilized to separate nuclear and cytoplasmic RNA from HCT116 or HT29 cells. Subsequently, RT‐qPCR was performed to analyze the RNA extracts from the cytoplasmic and nuclear fractions, with β‐actin and U6 being used as controls.

### 2.6 Western blot analysis

Total protein was isolated from HCT116 and HT29 cells using the Whole Cell Lysis Assay Kit (Keygen BioTECH). The protein concentration was determined, and 20 μL of total protein was mixed with SDS loading buffer, boiled for 5 min, and subjected to electrophoresis on a 10% SDS‐PAGE gel. The separated proteins were then transferred onto a PVDF membrane. After blocking and washing the membrane with PBS three times, the corresponding primary antibodies were added and incubated overnight at 4°C. Following three washes with PBS, the membrane was incubated with horseradish peroxidase‐conjugated secondary antibodies at room temperature for 1 h. After three additional washes with PBS, chemiluminescent detection was performed using the ECL Western Blotting Analysis System Kit. The gel was imaged using a gel imaging system, and the grayscale density values of the protein bands were analyzed. The antibodies used in this study, including E‐cadherin (ab181296), N‐cadherin (ab207608), Vimentin (ab13732), Snail (ab216347), Bax (Ab32503), Bcl‐2 (ab182858), Caspase3 (ab32351), Caspase 7 (ab255818), ERK1/2 (ab184699), pERK1/2 (ab201015), APC (ab40778), β‐catenin (ab32572), pβ‐catenin (ab75777), AXIN2 (ab109307), and GSK3β (ab32391), were obtained from Abcam (1:1000). GAPDH (ab9485) and Tubulin (ab7291) were also obtained from Abcam (1:5000). The protein band densities were quantified using Image J software version 1.8.0.

### 2.7 CCK‐8 assay

Cell proliferation was assessed using the Cell Counting Kit‐8 (APExBIO, USA). HCT116 or HT29 cells in the logarithmic growth phase were transferred to a 96‐well cell culture plate at a density of 1 × 10^4^ cells per well. Following a 12‐h incubation period for cell adhesion, the assay was initiated. CCK‐8 solution was added to each well at 24, 48, and 72 h of incubation, with a subsequent 1‐h incubation for color development. The absorbance values at 450 nm were measured using a microplate reader.

RETRACTED

### 2.8 Colony formation assay

The colony formation assay is used to assess long‐term cell proliferation. HCT116 and HT29 cells were seeded in six‐well plates at a density of 500 cells per well. When the cell colonies in each well exceeded 300, the culture dishes were removed. The cells were stained with 1% crystal violet at room temperature for 10 min, and the number of cell colonies was counted using an optical microscope (Olympus). Images were captured for documentation.

### 2.9 Cell cycle and apoptosis detection

1 × 10^6^ HCT116 or HT29 cells were cultured in McCoy 5A medium in a 12‐well plate for 24 h. The cells were then centrifuged at 300 × g for 5 min and washed twice with pre‐chilled 1 × PBS. Subsequently, the cells were fixed with pre‐chilled 70% ethanol (SolarBio) and kept at −20°C for at least 3 h. After centrifugation at 300 × *g* for 5 min, the cells were washed twice with pre‐chilled 1 × PBS. Next, the cells were incubated with 200 μL of MUSE Cell Cycle assay reagent (Muse™ Cell Cycle Kit, Millipore, USA) at room temperature, protected from light, for 30 min. Finally, cell cycle analysis was performed using the Muse Cell Analyzer, and the data were analyzed using the Muse_1500 Analysis software. In addition, following the instructions of the Muse™ Caspase‐3/7 Kit, 2 × 10^5^ cells/mL of HCT116 or HT29 cells were collected. 5 μL of Caspase‐3/7 working solution (prepared in a 1:8 PBS dilution) was added to 50 μL of cell suspension and incubated at 37°C for 30 min. Then, 150 μL of Caspase7‐ADD working solution (prepared in a 1:74 BA solution) was added and thoroughly mixed. The cells were incubated at room temperature, and protected from light, for 5 min. Cell apoptosis was detected using the Muse Cell Analyzer, and the data were analyzed using the Muse_1500 Analysis software.

### 2.10 Wound‐healing migration assay

A wound‐healing assay was performed on HCT116 and HT29 cells following various treatments. All cell cultures were dissociated into single‐cell suspensions in McCoy 5A medium, counted, and adjusted to a concentration of 6 × 105 cells/mL. Subsequently, 1 mL of the cell suspension was seeded into each well of a six‐well plate, supplemented with 1 mL of cell culture medium, and incubated at 37°C for 12 h. A sterile pipette tip was used to create a scratch wound on the cell monolayer, and images were captured under a microscope at *t* = 0 h to calculate the initial wound area. Images were also taken at 24 and 48 h (*t* = △h) to document the healing of the wounded monolayer due to migration in the scratched area. Images were captured using an inverted microscope equipped with a dynamic digital camera. The wound area was analyzed and calculated using ImageJ software. The remaining wound area percentage was determined as [(0 h area−△h area)/0 h area] × 100%.

RETRACTED

### 2.11 Cell migration and invasion analysis

Cell migration and invasion were evaluated using Transwell chambers equipped with an 8 μm membrane diameter. Before the assay, all cells underwent 2–3 passages and were subjected to 24 h of starvation. For the cell migration assessment, starved cells were collected in a serum‐free culture medium and adjusted to a concentration of 1.0 × 10^6^ cells/mL. Subsequently, 500 μL of 10% fetal bovine serum culture medium was introduced into the lower chamber of each Transwell, while 200 μL of serum‐free culture medium was placed in the upper chamber. The chambers were then incubated at 37°C with 5% carbon dioxide for 24 h. In the invasion assay, 200 μL of cells were introduced into the Transwell chambers that had been pre‐coated with matrix gel, following the identical procedure as the migration assay. After an incubation period, the chambers were extracted, rinsed twice with 1 × PBS, fixed with 4% paraformaldehyde for 5 min, rinsed again with 1 × PBS, and stained with 0.1% crystal violet solution. Subsequently, Images of cells that had migrated through the Transwell membrane or invaded the matrix gel were captured utilizing a microscope, and the cell areas within each group were assessed and computed using ImageJ software.

### 2.12 RNA pulldown and mass spectrometry analysis

The target sequence with a T7 promoter was amplified from the vector containing the target gene and purified as the probe for the RNA pulldown experiment. The sense strand with the T7 promoter was amplified by PCR and labeled as “Sense,” while the antisense strand with the T7 promoter was amplified by PCR and labeled as “Anti‐S.” The RNA was biotin‐labeled and then bound to streptavidin‐coated magnetic beads. The beads were washed twice with a Wash Buffer and placed on a magnetic rack to remove the wash buffer. Biotin‐labeled and denatured RNA was added to the beads and incubated at 4°C for 2 h with rotation. After incubation, the beads‐RNA complex was placed on the magnetic rack, and the supernatant was removed. The beads were washed twice with Wash Buffer. Cell lysis buffer (containing approximately 1 mg of protein) was added to the beads‐RNA complex, and an appropriate amount of RNase inhibitor was added to the lysis buffer. The mixture was incubated overnight at 4°C with rotation. The beads‐RNA‐protein complex was then retrieved from the overnight incubation, subjected to low‐speed centrifugation, placed on the magnetic rack, and the supernatant was removed. The beads were washed three times with Wash buffer. The sample was placed on the magnetic rack, and the supernatant was aspirated. Elution Buffer (40 μL) and 5× SDS protein loading buffer (10 μL) were added to the beads, and the mixture was incubated at 95°C with shaking for 10 min. After cooling to room temperature, the proteins were separated by 10% SDS‐PAGE and visualized by silver staining. For mass spectrometry analysis, an Orbitrap Exploris 480 mass spectrometer coupled with an EASY‐nLC 1200 liquid chromatography system was used for data acquisition. Peptide samples were dissolved in the loading buffer and loaded onto the analytical column (75 μm × 25 cm, C18, 1.9 μm, 100 Å) through an autosampler for separation. The mass spectrometry data were acquired in DDA mode, with each scan cycle consisting of one full MS scan followed by 20 MS/MS scans. The mass spectrometry data were analyzed using MaxQuant (V1.6.6) software with the Andromeda database search algorithm. The protein reference database used for the search was the human protein database in Uniprot.

RETRACTED

### 2.13 Animal tumorigenicity experiment

Resuscitated cultures of normal CRC HCT116 and HT29 cells, CCAT2 knockout cells, and cells overexpressing CCAT2 were used for subsequent animal experiments. Immunodeficient NOD‐SCID mice were acclimated for 1 week before the experiment. Log‐phase HCT116 and HT29 cells were collected. Cells were resuspended at a concentration of 1 × 10^7^ cells/100 μL per mouse and subcutaneously inoculated. Tumor size was measured twice a week, and the volume was calculated and recorded. Images were taken with a scale ruler for reference. Weight measurements were taken twice a week, and differences between different groups were recorded and analyzed. Tumor volume was calculated using the formula: tumor volume (mm^3^) = 0.5 × tumor length × (tumor width)^2^. The experimental animals were purchased from Hangzhou Ziyuan Experimental Animal Technology Co., Ltd., with the certificate number: 20230518Abzz0105000589.

### 2.14 Animal tumor metastasis experiment

After 1 week of acclimation, NOD‐SCID mice were used for the experiment. Normal colorectal cancer cells, CCAT2 knockout cells, and cells overexpressing CCAT2 were injected into the tail vein of immunodeficient mice to observe tumor metastasis. After 4 weeks, lung CT scans were performed to assess tumor metastasis. Samples were collected based on the CT results, and lung tissues were fixed for HE staining and scanning analysis.

RETRACTED

### 2.15 Statistical analysis

The comparison between two groups of samples was performed using an independent samples *t*‐test (T‐Test), while multiple group comparisons were conducted using one‐way analysis of variance (ANOVA). Data analysis was performed using SPSS, and graphing was done using GraphPad Prism. A significance level of *p* < 0.05 was considered statistically significant. Statistical charts and graphs were generated using GraphPad Prism 9 software.

## 3 RESULTS

### 3.1 The upregulation of lncRNA CCAT2 in CRC tissues and cell lines

It was investigated through the analysis of five CRC tissue samples and their corresponding adjacent normal tissue samples using transcriptome sequencing. A total of 5138 differentially expressed lncRNAs were identified, with 2351 being upregulated and 2787 downregulated (Figure 1A). Further analysis including pathway enrichment, co‐expression, and interaction network screening led to the selection of the top 50 lncRNAs for validation in CRC (Figure 1B). RT‐qPCR was utilized to assess the expression levels of CCAT2 in 101 CRC samples. The results demonstrated an upregulation of CCAT2 in CRC, with higher expression observed in 17 cases of metastatic CRC tissues compared to non‐metastatic CRC tissues (Figure 1C). Furthermore, in CRC cell lines HT29, HCT116, and SW620, CCAT2 expression exhibited an increasing trend in comparison to normal colonic epithelial cells NCM460 (Figure 1D). In conclusion, our findings indicate that CCAT2 is upregulated in CRC, particularly in metastatic CRC. Therefore, we believe that CCAT2 may play an important role in the development and metastasis of CRC.

**FIGURE 1:** Analysis and validation of the transcriptome sequencing results. (A) Volcano plot displaying the differentially expressed lncRNAs in tissue samples from five patients with CRC. The plot highlights the lncRNAs that are significantly upregulated (red dots) or downregulated (blue dots) in CRC. (B) The top 50 differentially expressed lncRNAs were selected from the sequencing results, the red‐highlighted part is the ID number of CCAT2 in the database. (C) The expression of CCAT2 was detected in tissue specimens from 101 patients with CRC and 17 patients with metastatic CRC patients. (D) The result of CCAT2 expression in CRC cells, ****p < 0.0001.

### 3.2 LncRNACCAT2 suppresses the proliferation, migration, and invasion of CRC cells

CRISPR/Cas9 gene knockout technology was utilized to target the CCAT2 gene in CRC cells HCT116 and HT29, with one upstream and one downstream target being designed (gRNA‐A1: TTACGGTTCATCACCAATAGTGG, gRNA‐A2: CACCAATAGTGGCAGAGGATGGG). Furthermore, a CCAT2 expression vector was constructed and transfected into HCT116 and HT29 cells. RT‐qPCR analysis indicated that CCAT2 expression was not detectable in the CCAT2 knockout group (CCAT2‐KO), significantly increased in the CCAT2 overexpression group (CCAT2‐OE), and restored in the CCAT2 knockout cells transfected with the expression vector (CCAT2‐KO+OE) (Figure 2A). Cell proliferation was evaluated using the CCK‐8 assay, revealing a decrease in proliferation capacity in CCAT2‐KO cells and an increase in proliferation in CCAT2‐OE cells. the CCAT2‐KO+OE group exhibited enhancedcell proliferation compared to the CCAT2‐KO group (Figure 2B,C). Additionally, the colony formation assay indicated a decrease in the number of cell colonies in the CCAT2‐KO group compared to the control group and an increase in the CCAT2‐OE group. In the CCAT2‐KO+OE group, there was an increase in the number of cell colonies compared to the CCAT2‐KO group (Figure 2D and supplementary S1A). The scratch wound healing assay demonstrated that CCAT2‐KO cells exhibited decreased migration speed, whereas CCAT2‐OE cells displayed increased migration speed. In the CCAT2‐KO+OE group, cell migration speed was elevated compared to the CCAT2‐KO group (Figure 2E and supplementary S1B).

RETRACTED

**FIGURE 2:** Effects of CCAT2 knockout and overexpression on proliferation, migration, and invasion of CRC cells. (A) RT‐qPCR results show the expression levels of CCAT2 in CRC cells with CCAT2 knockout and overexpression. (B, C) CCK8 assay results demonstrate the proliferation of HCT116 and HT29 cells with CCAT2 knockout and overexpression, respectively. (D) Results of cell cloning experiments to assess the effect of CCAT2 knockout and overexpression on colony formation in HCT116 cells. (E) Wound healing scratch assay to evaluate the migration ability of CRC cells with CCAT2 knockout and overexpression. (F, G) Transwell assays were performed to assess the migratory and invasive abilities of HCT116 and HT29 cells with CCAT2 knockout and overexpression, **p < 0.01, ***p < 0.001, ****p < 0.0001.

Migration and invasion capabilities were evaluated using 8 μm Transwell chambers and Matrigel invasion assays, respectively. The findings indicated that CCAT2‐KO cells had significantly diminished migration and invasion abilities, while CCAT2‐OE cells showed enhanced capabilities. In the CCAT2‐KO+OE group, both migration and invasion abilities were augmented compared to the CCAT2‐KO group. Statistical analysis revealed significant differences among the groups (Figure 2F,G). We also examined the expression of epithelial‐mesenchymal transition (EMT) markers in HCT116 and HT29 cells treated with varying interventions demonstrated distinct patterns. Specifically in the CCAT2‐KO group, there was an increase in the expression of epithelial marker E‐cadherin, accompanied by a decrease in the expression of mesenchymal markers N‐cadherin, Vimentin, and Snail. Conversely, in the CCAT2‐OE group, a decrease in E‐cadherin expression was observed alongside an increase in N‐cadherin, Vimentin, and Snail expression. In the CCAT2‐KO+OE group, there was a decrease in the expression of E‐cadherin compared to the CCAT2‐KO group, while the expression of N‐cadherin, Vimentin, and Snail was increased (Figure 3A and supplementary S1C). These results indicate that the knockout of the CCAT2 gene suppresses the proliferation, migration, and invasion capabilities of CRC cells.

RETRACTED

**FIGURE 3:** Effects of CCAT2 knockout and overexpression on apoptosis and cell cycle regulation in CRC cells. (A) Western blot analysis of EMT marker protein expression in HCT116 cells after CCAT2 knockout and overexpression. (B) Results of functional enrichment analysis of CCAT2 target genes. (C) Apoptosis assay results of HCT116 cells with CCAT2 knockout and overexpression. (D, E) Detection of apoptosis‐related protein expression in CRC cells with CCAT2 knockout and overexpression. (F) Results of cell cycle distribution analysis and statistical analysis in HCT116 cells after CCAT2 knockout and overexpression, *p < 0.05, **p < 0.01, ***p < 0.001, ****p < 0.0001, ns indicates no statistically significant difference.

### 3.3 LncRNA CCAT2 suppresses apoptosis in CRC cells

According to the anticipated outcomes obtained from online databases, it was determined that CCAT2 plays a role in various biological processes and metabolic pathways, such as apoptosis, cell cycle regulation, and signaling pathways like ERK and Wnt (Figure 3B). To delve deeper into the influence of CCAT2 on apoptosis in colorectal cancer cells, the Millipore Muse™ Caspase‐3/7 Kit was utilized for detection. The findings revealed a rise in apoptotic cell count in the CCAT2 knockout group, whereas a decline was noted in the CCAT2 overexpression group. In the CCAT2‐KO+OE group, a reduction in the number of apoptotic cells was observed, suggesting that CCAT2 knockout may enhance apoptosis, whereas CCAT2 itself may inhibit apoptosis in CRC cells (Figure 3C and supplementary S1E).

Additionally, the analysis of apoptosis‐related protein expression revealed in the CCAT2‐KO group, there was an increase in the levels of Bax, Caspase3, and Caspase7 proteins, accompanied by a decrease in BCL2 protein expression. Conversely, in the CCAT2‐OE group, there was a decrease in the levels of Bax, Caspase3, and Caspase7 proteins, along with an increase in BCL2 protein expression. In the CCAT2‐KO+OE group, a slight downregulation in the expression of Bax, Caspase3, and Caspase7 proteins was observed compared to the CCAT2‐KO group, providing additional validation to our conclusion (Figure 3D,E, and supplementary S1D). Our study indicates that the knockout of the CCAT2 gene can enhance apoptosis in CRC cells, leading to alterations in the expression of apoptosis‐related proteins.

RETRACTED

### 3.4 Knockout of the CCAT2 gene promotes G2/M phase prolongation in CRC cells

We used the Muse™ Cell Cycle Kit to examine the cell cycle of HCT116 and HT29 cells and found that knockout of the CCAT2 gene can promote G2/M phase prolongation in CRC cells. Specifically, compared to the control group, the proportion of cells in the G2/M phase increased in the CCAT2 knockout group, while the proportion of cells in the G0/G1 phase decreased (Figure 3F and supplementary S1F). These results indicate that knockout of the CCAT2 gene leads to G2/M phase prolongation in CRC cells, thereby inhibiting cell proliferation.

### 3.5 CCAT2 regulates the proliferation and metastasis of CRC through influence on the ERK and Wnt signaling pathways

Through analysis of the predicted target genes of CCAT2, its role in modulating these pathways was confirmed. Experimental validation of this prediction involved the examination of ERK protein expression and phosphorylation levels of ERK, which revealed that knockout of the CCAT2 gene led to inhibition of ERK phosphorylation of ERK (Figure 4A,B). Furthermore, the expression of key proteins in the Wnt signaling pathway, such as β‐catenin, APC, AXIN2, and GSK3β, was assessed to further elucidate the impact of CCAT2 on these signaling pathways. The findings indicate that in the CCAT2‐KO group, there was an upregulation in the expression of APC, AXIN2, and GSK3β proteins, alongside a downregulation in the expression of β‐catenin protein. Additionally, there was an increase in the expression of phosphorylated β‐catenin. Conversely, in the CCAT2 overexpression group, there was a downregulation in the expression of APC, AXIN2, and GSK3β proteins, while there was an upregulation in the expression of β‐catenin protein and a decrease in the expression of phosphorylated β‐catenin (Figure 4C,D). These results indicate that the knockout of the CCAT2 leads to the suppression of both the Wnt and ERK signaling pathways, thereby influencing the proliferation and metastasis of CRC.

**FIGURE 4:** Expression of ERK and Wnt pathway‐related proteins in CRC cells with knockout and overexpression of CCAT2, and analysis of subcellular localization of CCAT2 in CRC cells. (A, B) Expression and statistical analysis of ERK and pERK levels in HCT116 and HT29 cells with CCAT2 knockout and overexpression, respectively. (C, D) Expression and statistical analysis of Wnt signaling pathway‐related proteins, including β‐catenin and its phosphorylation status, APC, AXIN2, and GSK3β, in HCT116 and HT29 cells with CCAT2 knockout and overexpression. (E, F) Subcellular localization of CCAT2 in HCT116 and HT29 cells, *p < 0.05, **p < 0.01, ***p < 0.001, ****p < 0.0001.

RETRACTED

### 3.6 LncRNA CCAT2 promotes tumor growth and metastasis in CRC cells in vivo

In vivo, experiments involving the injection of HCT116 and HT29 cells into immunodeficient mice revealed that mice injected with CCAT2‐KO cells exhibited significantly smaller tumor volumes and masses compared to those control cells. Administered with CCAT2‐KO+OE cells exhibited increased tumor volumes and masses in comparison to both the control group and the CCAT2‐KO group (Figure 5A,E). Furthermore, tumor metastasis was evaluated by intravenously injecting cells from each group into mice and monitoring the development of metastatic lesions. Following a 4‐week observation period, CT scan findings revealed a decreased number of lung tumor foci in the CCAT2‐KO group, whereas mice in the CCAT2‐KO+OE group displayed a higher incidence of lung tumor foci (Figure 5B,F). Further analysis of the mice revealed minimal tumor formation in the lungs of mice administered with CCAT2‐KO cells, in contrast to both the control group and CCAT2‐K+ OE group, which exhibited tumor formation. Notably, the CCAT2‐KO+OE group displayed a higher incidence of tumors (Figure 5C,G). Histological examination using hematoxylin and eosin staining confirmed the presence of tumors in the lungs of mice injected with normal CRC cells, whereas mice injected with CCAT2‐KO cells exhibited limited tumor formation. Additionally, the CCAT2‐KO+OE group displayed larger tumor areas in the lungs (Figure 5D,H). The findings from the in vivo experiments involving mice indicate that the injection of CCAT2‐KO cells leads to reduced tumor volumes and masses, whereas the injection of CCAT2‐KO+OE cells results in increased tumor volumes and masses. Additionally, CCAT2‐KO cells demonstrate metastatic potential, while CCAT2‐KO+OE cells exhibit heightened metastatic potential.

**FIGURE 5:** Results of in vivo tumor formation and metastasis experiments using CCAT2 knockout and post‐knockout overexpressing CRC cells in mice. (A, E) Subcutaneous tumor formation in immunodeficient mice injected with CCAT2 knockout and post‐knockout overexpressing CRC cells. Statistical analysis of tumor growth is also presented, providing insights into the role of CCAT2 in tumor formation in vivo. (B, F) CT scan results show lung metastases from tumors formed by intravenous injection of CRC cells into the tail vein of immunodeficient mice. (C, G) Metastasis results of CCAT2 knockout and post‐knockout overexpressing CRC cells in mouse lungs. (D, H) Hematoxylin and eosin (HE) staining results of mouse lung tissue, highlighting the presence of metastatic lesions, *p < 0.05, **p < 0.01, ***p < 0.001.

RETRACTED

### 3.7 Identification of CCAT2 binding with GNB2 protein through RNA‐pulldown and mass spectrometry analysis

A specific probe was designed using the CCAT2 sequence, and RNA‐pulldown experiments were conducted to detect proteins binding to CCAT2. Proteins binding to CCAT2 were observed using SDS‐PAGE electrophoresis and silver staining (Figure 6A). Proteins binding to CCAT2 were identified through mass spectrometry analysis, with specific binding proteins identified through screening (Figure 6B,C). Further analysis was conducted by performing RNA sequencing on HCT116 cells with CCAT2 knockout, cells expressing CCAT2, and the CCAT2 pulldown protein mass spectrometry results. Venn diagrams identify differentially expressed genes in each group, resulting in the identification of three differentially expressed genes, which are GNB2, RPL17, and CSTA (Figure 6D,E). To confirm the findings, Western blot analysis was utilized to identify the presence of protein in the RNA‐pulldown samples. The data revealed the detection of GNB2 protein in both in the Input and CCAT2 pulldown groups, but not in the control group (Figure 6F). These findings indicate that CCAT2 can bind and interact with GNB2 protein.

**FIGURE 6:** CCAT target protein screening and validation results. (A) SDS‐page gel electrophoresis with silver staining showing the result of CCAT2 RNA pulldown. (B) Heatmap depicting the detection of CCAT2 probe pull‐down proteins using mass spectrometry. (C) CCAT2 probe pull‐down proteins with significant differences in protein distribution. (D) Venn diagram showing the overlap between the sequencing results of CCAT2 knockout and overexpression and the mass spectrometry analysis of CCAT2 RNA pulldown. (E) Sequencing results of HT29 cells with CCAT2 knockdown and overexpression, reveal the differential expression of genes. (F) Western blot validation of the RNA pulldown results, confirming the interaction between CCAT2 and specific target proteins. (G) Immunohistochemical results show the expression of the CCAT2 target protein GNB2 in CRC tissues. (H) Western blot detection of GNB2 expression in CRC cells, **p < 0.01, ****p < 0.0001.

RETRACTED

### 3.8 CCAT2 positively regulates the expression of GNB2 in CRC cell

Immunohistochemistry was conducted to assess the expression levels of GNB2 protein in 40 CRC tissues and their corresponding adjacent non‐cancerous tissues. The results demonstrated a significant upregulation of GNB2 protein expression in CRC tissues compared to adjacent non‐cancerous tissues. Moreover, the results from Western blot analysis indicated an increase in GNB2 expression in CRC cells HCT116 and HT29 compared to normal colonic epithelial cells NCM460 (Figure 6G,H). Transcriptome sequencing analysis also confirmed the upregulation of both CCAT2 and GNB2 in CRC tissues (Figure 7A). Subsequent RT‐qPCR analysis demonstrated elevated GNB2 expression in 117 CRC tissues, particularly in metastatic CRC tissues. Co‐expression analysis revealed a positive relationship between CCAT2 and GNB2 in CRC tissues (Figure 7B,C). Western blot analysis demonstrated downregulated expression of GNB2 in CCAT2‐KO cells, upregulated expression in CCAT2‐OE cells, and higher expression in CCAT2‐KO+OE cells compared to the control group (Figure 7D). These findings indicate that CCAT2 positively regulates the expression of GNB2 in CRC and that there is a positive co‐expression relationship between the two in CRC tissues. These findings further support the important role of CCAT2 in CRC development and provide clues for further investigation into the functions of CCAT2 and GNB2.

**FIGURE 7:** GNB2 expression analysis and results of proliferation, migration, and invasion of CRC cells with CCAT2 knockout and GNB2 overexpression. (A) The transcriptome sequencing results showing lncRNA and mRNA co‐expression analysis. (B) RT‐qPCR validation of GNB2 expression in CRC and metastases CRC tissues. (C) Results of correlation analysis between CCAT2 and GNB2 expression in CRC. (D) Western blot validation of GNB2 expression in CRC cells with CCAT2 knockout and overexpression. (E) Detection of the effect of GNB2 overexpression on GNB2 expression by transfecting CRC cells with a GNB2 overexpression vector. (F) Results of cell cloning experiments to assess community formation in HCT116 cells with CCAT2 knockout and GNB2 overexpression. (G) Transwell assays were performed to detect the migratory and invasion abilities of CRC cells with CCAT2 knockout and GNB2 overexpression, **p < 0.01, ***p < 0.001, ****p < 0.0001.

### 3.9 CCAT2 promotes CRC cell proliferation, migration, and invasion by regulating GNB2

An expression vector for GNB2 (GNB2‐OE) was constructed and its expression in CRC cells through experiments. The findings indicated a decrease in GNB2 expression in the CCAT2‐KO group, whereas in the GNB2‐OE group, GNB2 expression was elevated relative to the control group. Additionally, the overexpression of GNB2 following CCAT2 knockout (CCAT2‐KO+GNB2‐OE) resulted in a higher level of GNB2 expression compared to the CCAT2‐KO group (Figure 7E). Clonogenic assays demonstrated an increased proliferative capacity in GNB2‐OE cells in comparison to the control group. Furthermore, the study found that the proliferative capacity of CRC cells was significantly increased in the CCAT2‐KO+GNB2‐OE group compared to the CCAT2‐KO group (Figure 7F and supplementary S2A). To evaluate the migration ability of CRC cells, scratch wound healing assays were conducted in the CCAT2‐KO, GNB2‐OE, and CCAT2‐KO+GNB2‐OE treatment groups. The results indicated that CCAT2‐KO cells exhibited slower migration, while GNB2‐OE cells showed faster migration. Interestingly, in the CCAT2‐KO+GNB2‐OE group, there was a notable increase in cell migration speed compared to the CCAT2‐KO group (supplementary S2B,C).

RETRACTED

Transwell assays were utilized to assess the migratory and invasive CRC cells in the CCAT2‐KO, GNB2‐OE, and CCAT2‐KO+GNB2‐OE treatment groups. The findings indicated diminished migration and invasion capacities in the CCAT2‐KO group, whereas the GNB2‐OE group displayed notably enhanced migration and invasion capabilities. In the CCAT2‐KO+GNB2‐OE treatment group, cell migration and invasion rates were elevated compared to the CCAT2‐KO group (Figure 7G). Additionally, the expression levels of epithelial‐mesenchymal transition (EMT) marker proteins in HCT116 and HT29 cells of each treatment group. The findings indicate that the CCAT2‐KO group exhibited increased expression of the epithelial marker E‐cadherin, alongside decreased expression of the mesenchymal markers N‐cadherin, Vimentin, and Snail. Conversely, the GNB2‐OE group displayed decreased E‐cadherin expression and increased expression of N‐cadherin, Vimentin, and Snail. In the CCAT2‐KO+GNB2‐OE group, E‐cadherin expression was reduced, while N‐cadherin, Vimentin, and Snail expression was elevated, effectively, reversing the impact of CCAT2 knockout (Figure 8A,B, and supplementary S3G). The results of our study indicate that CCAT2 plays a regulatory role in promoting CRC.cell proliferation, migration, and invasion, by modulating GNB2 expression, as well as influencing the expression of EMT marker proteins.

**FIGURE 8:** Effects of CCAT2 knockout and GNB2 overexpression on EMT proteins, apoptosis, cell cycle, ERK, and Wnt pathway proteins in CRC cells. (A, B) Western blot analysis of EMT marker protein expression and statistical analysis in CRC cells after CCAT2 knockout and GNB2 overexpression. (C) Apoptosis assay results in HCT116 cells with CCAT2 knockout and GNB2 overexpression. (D) Results of cell cycle distribution analysis and statistical analysis in HCT116 cells after CCAT2 knockout and GNB2 overexpression. (E, F) Detection of apoptosis‐related protein expression in CRC cells with CCAT2 knockout and GNB2 overexpression in HCT116 cells. (G, H) Expression and statistical analysis of ERK and pERK levels in HCT116 and HT29 cells with CCAT2 knockout and GNB2 overexpression. (I, J) Expression and statistical analysis of Wnt signaling pathway‐related proteins, including β‐catenin and its phosphorylation status, APC, AXIN2, and GSK3β, in HCT116, and HT29 cells with CCAT2 knockout and GNB2 overexpression, *p < 0.05, **p < 0.01, ***p < 0.001, ****p < 0.0001, ns indicates no statistically significant difference.

RETRACTED

### 3.10 CCAT2 regulates apoptosis of CRC cells through the modulation of GNB2

Apoptosis of CRC cells was evaluated in treatment groups with CCAT2‐KO, GNB2‐OE, and CCAT2‐KO+GNB2‐OE using the Millipore Muse™ Caspase‐3/7 Kit. The findings indicated a higher number of apoptotic cells in the CCAT2‐KO group compared to the control group, whereas a decrease in apoptotic cells was observed in the GNB2‐OE group. In the CCAT2‐KO+GNB2‐OE group, the number of apoptotic cells decreased in comparison to the CCAT2‐KO group (Figure 8C and supplementary S2D). Furthermore, the expression of apoptosis‐related proteins. The findings demonstrated a significant increase in the expression levels of Bax, Caspase3, and Caspase7 proteins, along with a decrease in BCL2 protein in the CCAT2‐KO group. Conversely, in the GNB2‐OE group, there was a decrease in the expression of Bax, Caspase3, and Caspase7 proteins accompanied by an increase in BCL2 protein expression. Additionally, in the CCAT2‐KO + GNB2‐OE group, the expression levels of Bax, Caspase3, and Caspase7 proteins were also decreased compared to the CCAT2‐KO group (Figure 8E,F, and supplementary S3H). Our findings suggest that CCAT2 is involved in the regulation of CRC cells apoptosis through the modulation of GNB2 expression and the expression of apoptosis‐related proteins.

### 3.11 CCAT2 is involved in the regulation of the cell cycle distribution of CRC cells by modulating GNB2

The cell cycle distribution of HCT116 and HT29 cells was analyzed using the Muse™ Cell Cycle Kit. The results showed an increase in G2M phase cells and a decrease in G0G1 phase cells in the CCAT2‐KO group compared to the control group. Furthermore, in the CCAT2‐KO+GNB2‐OE group, the proportion of G2M phase cells was reduced compared to the CCAT2‐KO group (Figure 8D and supplementary S2E). The se alterations in cell cycle distribution are associated with the regulation of CCAT2 and GNB2.

RETRACTED

### 3.12 CCAT2 regulates CRC proliferation and metastasis through the modulation of the ERK and Wnt signaling pathways by GNB2

The study examined the role of GNB2 in the ERK and Wnt signaling pathways by constructing GNB2 interference plasmids and The study examined the role of GNB2 expression levels in GNB2‐si‐1 and GNB2‐si‐2 interference plasmids. The findings demonstrated a substantial decrease in GNB2 expression in both GNB2‐si‐1 and GNB2‐si‐2 interference plasmids (supplementary S3A,B). Our study revealed that modulation of GNB2 expression results in the inhibition of ERK phosphorylation levels and a simultaneous increase in β‐catenin phosphorylation levels, ultimately leading to a decrease in β‐catenin expression. This observation aligns with the effects observed following CCAT2 knockout, suggesting a regulatory role for CCAT2. (supplementary S3C–F). Subsequent analysis of ERK and phosphorylated ERK proteins indicated that CCAT2‐KO decreased the phosphorylation level of ERK, whereas GNB2‐OE elevated the phosphorylation level of ERK. In the CCAT2‐KO+GNB2‐OE group, the phosphorylation level of ERK was increased compared to the CCAT2‐KO group (Figure 8G,H, and supplementary S3I). Furthermore, we investigated the key proteins involved in the Wnt signaling pathway. The findings demonstrated that in the GNB2‐OE group, the protein expression of APC, AXIN2, and GSK3β was reduced, while β‐catenin protein expression was enhanced, and the expression of phosphorylated β‐catenin was decreased. In the CCAT2‐KO+GNB2‐OE group, the protein expression levels of APC, AXIN2, and GSK3β were found to be decreased in comparison to the CCAT2‐KO group Conversely, the expression of β‐catenin protein was increased, while the expression of phosphorylated β‐catenin was decreased. These results indicate that the overexpression of GNB2 can counteract the regulatory impacts of CCAT2 knockout (Figure 8I,J, and supplementary S2J). These research findings demonstrate that knocking out CCAT2 inhibits the activity of the Wnt and ERK signaling pathways while overexpressing GNB2 produces the opposite effect. Moreover, the upregulation of GNB2 in CCAT2‐deficient cells has been found to mitigate the consequences of CCAT2 deletion. This finding provides further evidence that CCAT2 modulates the functionality of the Wnt and ERK signaling pathways through its regulation of GNB2 protein expression.

## 4 DISCUSSION

Based on the results of our study, it has been determined that lncRNA CCAT2 exhibits upregulation in CRC, especially in cases of metastatic CRC. In vitro cell experiments have demonstrated that the deletion of CCAT2 can inhibit the proliferation, migration, and invasion of CRC cells while enhancing cell apoptosis. These findings imply a significant involvement of CCAT2 in the pathogenesis of CRC. Additional experimental data suggests that CCAT2 interacts with and modulates the GNB2 protein, thereby impacting the proliferation and metastasis of CRC. Utilizing RNA‐pulldown in conjunction with protein mass spectrometry, we have successfully elucidated the interaction between CCAT2 and GNB2 protein, as along with the regulatory GNB2 expression. Furthermore, our investigation has unveiled that alterations in GNB2 protein mediated by CCAT2 have profound implications on the ERK and Wnt signaling pathways, ultimately fostering the proliferation and metastasis of CRC. The intricate regulatory mechanisms governing the proliferation and metastasis of CRC involve a multitude of factors, with the ERK and Wnt signaling pathways serving as pivotal components. The results of our study indicate that CCAT2 modulates the ERK and Wnt signaling pathways through its regulation of GNB2 protein expression. Specifically, CCAT2 knockout leads to decreased ERK phosphorylation and inhibition of Wnt signaling activity, whereas GNB2 overexpression has the opposite effect. Additionally, the overexpression of GNB2 in CCAT2 knockout cells can reverse the effects induced by CCAT2 knockout.

RETRACTED

CCAT2 is a lncRNA and has been identified as an oncogenic factor in multiple tumor types. Studies have demonstrated that CCAT2 is upregulated in small‐cell lung cancer patients and is associated with poor prognosis, acting as an independent predictor of poor outcomes.^15^ In non‐small cell lung cancer, CCAT2 facilitates tumorigenesis through the upregulation of Pokemon, potentially involving the Pokemon‐related gene p21.^16^ Additionally, in colorectal cancer patients, elevated levels of CCAT2 are strongly associated with advanced tumor progression and poor prognosis.^11^ Hence, the upregulation of CCAT2 may serve as a promising diagnostic biomarker for CRC and an independent prognostic factor for patient outcomes. Furthermore, elevated levels of CCAT2 have been detected in ovarian cancer tissues, correlating with decreased overall and disease‐free survival rates, indicating a poor prognosis.^17^ In CRC, we have observed upregulated expression of CCAT2, particularly in metastatic CRC. Thus, CCAT2 can be utilized as an auxiliary indicator for prognostic evaluation or a predictive factor for individualized treatment, aiding in guiding treatment decisions for CRC patients. Therefore, the overexpression of CCAT2 is significantly linked to poor prognosis in various tumors. In CRC, increased expression of CCAT2 may play a crucial role in prognostic assessment and personalized treatment prediction. Further exploration of the functions and mechanisms of CCAT2 will enhance comprehension of its involvement in tumor progression, offering novel therapeutic targets and strategies for managing CRC.

RETRACTED

CCAT2 has been extensively studied in various tumors, primarily in relation to tumor diagnosis and prognosis, although its specific mechanisms of action remain unclear. Some studies have reported on the regulatory mechanisms and functions of CCAT2 in different tumors. For example, in gastric cancer research, CCAT2 has been shown to interact with epithelial splicing regulatory protein 1 (ESRP1), leading to the upregulation of CD44v6 expression and mediating alternative splicing of CD44. This regulatory mechanism promotes the progression of gastric cancer, and in vitro and in vivo experiments have confirmed the oncogenic role of the CCAT2/ESRP1/CD44 axis in promoting malignant behavior.^18^ In neuroblastoma, CCAT2 expression has been found to inhibit cell proliferation and promote apoptosis, providing a foundation for the treatment of neuroblastoma. In prostate cancer, CCAT2 has been shown to promote cell proliferation and invasion by regulating the Wnt/β‐catenin signaling pathway.^19^ CCAT2 may play a critical role in the progression of prostate cancer and could serve as a therapeutic target for the disease.^20^ CCAT2 regulates the cell cycle, migration, and apoptosis in MCF7‐R cells through the hsa‐miR‐145‐5p/AKT3/mTOR axis. Additionally, CCAT2 enhances the sensitivity of breast cancer cells (MCF7) to tamoxifen.^21^ In colon cancer cells, the overexpression of CCAT2 promotes chromosomal instability and carcinogenesis by stabilizing and inducing the expression of the aurora kinase B activator BOP1.^22^ This provides a possibility for the development of therapeutic strategies targeting this pathway for patients with microsatellite‐stable colorectal tumors. CCAT2 plays important roles in various tumors, involving multiple signaling pathways and molecular regulations. However, further in‐depth research is needed to better understand the mechanisms of action of CCAT2 and its potential clinical applications in tumor development.

The Wnt signaling pathway and the ERK signaling pathway play crucial roles in the occurrence and development of CRC. The Wnt signaling pathway is closely associated with various aspects of cancer cells, including proliferation, apoptosis, autophagy, metabolism, inflammation, and immunity, microenvironment, drug resistance, ion channels, heterogeneity, as well as EMT/migration/invasion/metastasis.^23^, ^24^, ^25^, ^26^ Drugs and molecular agents targeting the Wnt signaling pathway have been developed and widely applied in the treatment of CRC. Wnt inhibitors are commonly used in clinical practice for the treatment of CRC.^27^ The Wnt signaling pathway is a complex regulatory network that participates in multiple physiological processes of CRC, including carcinogenesis, progression, prognosis, invasion, and metastasis.^28^ In the field of cancer research, lncRNAs have been identified as key regulators of tumorigenesis, metastasis, and treatment outcomes through their modulation of the Wnt signaling pathway. For instance, LINC00669 has been shown to activate the Wnt/β‐catenin pathway, leading to enhanced growth of lung adenocarcinoma and impacting patient prognosis.^29^ Similarly, AFAP1‐AS1 has been found to drive epithelial‐mesenchymal transition and tumorigenesis in triple‐negative breast cancer by modulating the Wnt/β‐catenin signaling cascade.^30^ Conversely, FOXO1‐induced LyPLAL1‐DT has been demonstrated to impede the progression of triple‐negative breast cancer by disrupting the hnRNPK/β‐catenin complex.^31^ In the context of colorectal cancer, numerous studies have elucidated the involvement of long non‐coding RNAs (lncRNAs) in modulating the Wnt signaling pathway. For example, lncRNA RMST has been shown to impede the progression of colorectal cancer by competitively binding to the miR‐27a‐3p/RXRα axis, thereby inhibiting Wnt signaling.^32^ Additionally, lncRNA STEAP3‐AS1 has been implicated in promoting colorectal cancer progression through the STEAP3‐AS1/STEAP3/Wnt/β‐catenin axis, suggesting the potential utility of these lncRNAs as diagnostic biomarkers or therapeutic targets for improving colorectal cancer treatment.^33^ The ERK pathway is one of the most important MAPK pathways. It is activated by phosphorylation of MEK, which in turn is activated by phosphorylation of Raf.^34^ The ERK/MAPK pathway is also one of the most commonly affected pathways in cancer.^35^, ^36^ In recent years, studies have shown that long non‐coding RNAs (lncRNAs) play important roles in the regulation of signaling pathways in cancer, including the ERK pathway.^37^, ^38^ Our research findings indicate that CCAT2 can simultaneously regulate the ERK and Wnt signaling pathways, which is of significant importance in CRC research. The Wnt signaling pathway and the ERK signaling pathway play important roles in CRC research. In‐depth studies of these two signaling pathways contribute to a better understanding of the mechanisms underlying CRC development and provide new targets and strategies for the treatment and prognosis evaluation of this disease. The dual regulation of CCAT2 in these two signaling pathways offers a new perspective and potential for CRC research.

RETRACTED

Our research has demonstrated that the guanine nucleotide‐binding protein 2 (GNB2) is upregulated in CRC tissues and shows a co‐expression correlation with CCAT2. Knockdown of CCAT2 leads to a decrease in GNB2 expression, and our RNA‐pulldown technique combined with proteomic analysis has identified their interaction. Additionally, the overexpression of GNB2 in CCAT2‐knockout cells restores cell proliferation, migration, and invasion capabilities while suppressing apoptosis. These results indicate that CCAT2 interacts with GNB2 to regulate the proliferation and metastasis of CRC. The underlying mechanism entails the modulation of the ERK and Wnt signaling pathways, with a comprehensive analysis across 23 cancer types and significant upregulation of GNB2.^39^ Particularly, heightened expression of GNB2 in hepatocellular carcinoma (LIHC) and colorectal adenocarcinoma (READ) correlates with diminished overall survival (OS), underscoring the pivotal, role of GNB2 in the tumorigenesis of LIHC and READ. GNB2 has been identified as a common potential biomarker for LIHC and READ. Further analysis has revealed the involvement of GNB2 in promoter methylation, tumor purity, CD8+ T cell infiltration, genetic alterations, and chemotherapy drugs. Studies have shown that miR‐142‐3p improves resistance to paclitaxel (PTX) by targeting GNB2, and downregulation of GNB2 activates the AKT–mTOR pathway.^13^ GNB2 serves as an important target of miR‐142‐3p in inhibiting autophagy, providing new insights for improving PTX treatment in breast cancer. Limited research has been conducted on GNB2 in CRC, and its specific mechanisms of action remain unclear. Our research demonstrates the influence of CCAT2 on ERK and Wnt signaling pathways by modulating GNB2, presenting a novel discovery in the mechanisms of proliferation, metastasis, and apoptosis in CRC. CCAT2 has the potential to be a valuable biomarker for the detection, management, and prediction of outcomes in CRC. However, limited research has been conducted on the involvement of GNB2 in CRC, necessitating further investigation into its mechanism of action. Additionally, this study fails to elucidate the specific binding sequence between lncRNA CCAT2 and GNB2, as well as the core sequence through which CCAT2 operates. Despite diligent research efforts, a definitive target sequence remains elusive. Clarifying the functional core sequence of CCAT2 is crucial for a comprehensive exploration of its molecular function, such as designing targeted therapies based on functional sequences.

In summary, the results of our study have elucidated the pivotal function of the lncRNA CCAT2 in the proliferation and metastasis of CRC. Through its interaction with GNB2, CCAT2 modulates the ERK and Wnt signaling pathways, thereby accelerating the progression of CRC. This discovery provides new clues for a deeper understanding of the pathogenesis of CRC and offers potential targets for the development of therapeutic strategies targeting CCAT2 and GNB2. However, further studies are needed to explore the detailed regulatory mechanisms of CCAT2 and GNB2 in CRC and to validate their potential clinical applications.

RETRACTED

## AUTHOR CONTRIBUTIONS

**Jinhai Tian:** Investigation (lead); methodology (supporting); project administration (equal); validation (lead); writing – original draft (lead). **Xu Cao:** Data curation (equal); formal analysis (equal); methodology (equal); software (equal). **Zongying Jiang:** Data curation (equal); methodology (equal); resources (equal); software (equal); validation (equal). **Jia Wang:** Data curation (equal); supervision (equal); validation (equal); visualization (equal). **Wan Fan:** Formal analysis (equal); methodology (equal); software (equal). **Shaoting Zhang:** Formal analysis (equal); methodology (equal); resources (equal); software (equal); validation (equal). **Sien Zhao:** Data curation (equal); formal analysis (equal); methodology (equal). **Jianmin Sun:** Conceptualization (supporting); investigation (supporting); project administration (supporting); resources (supporting); writing – original draft (equal).

## FUNDING INFORMATION

Key Research and Development Program Project of Ningxia province, Grant/Award Number: 2021BEG03089, Natural Science Foundation of Ningxia province, Grant/Award Number: 2021AAC03380 and The Science Research Project of Ningxia Medical University, Grant/Award Number: XM2018099.

## CONFLICT OF INTEREST STATEMENT

The authors declare no conflict of interest.

## Supporting information


**Data S1.** Effects of CCAT2 knockout and overexpression on proliferation, migration, invasion, apoptosis, and cell cycle in CRC cells. (A) Results of cell cloning experiments to assess community formation in HT29 cells with CCAT2 knockout and overexpression. (B) Wound healing scratch assay to detect the migration ability of HT29 cells with CCAT2 knockout and overexpression. (C) Western blot analysis of EMT marker protein expression and statistical analysis in HT29 cells after CCAT2 knockout and overexpression. (D) Statistical analysis of Western blot results, providing quantitative information on the expression levels of EMT marker proteins in HT29 cells with CCAT2 knockout and overexpression. (E) Apoptosis assay results in HT29 cells with CCAT2 knockout and overexpression. (F) Results of cell cycle distribution analysis and statistical analysis in HT29 cells after CCAT2 knockout and overexpression, *p < 0.05, **p < 0.01, ***p < 0.001, ****p < 0.0001, ns indicates no statistically significant difference.

RETRACTED

**Data S2.** Effects of CCAT2 knockout and GNB2 overexpression on proliferation, migration, invasion, apoptosis, and cell cycle in CRC cells. (A) Results of cell cloning experiments to assess community formation in HT29 cells with CCAT2 knockout and GNB2 overexpression. (B, C) Wound healing scratch assay to detect the migration ability of HT29 cells with CCAT2 knockout and GNB2 overexpression. (D) Apoptosis assay results in HT29 cells with CCAT2 knockout and GNB2 overexpression. (E) Results of cell cycle distribution analysis and statistical analysis in HT29 cells after CCAT2 knockout and GNB2 overexpression, *p < 0.05, **p < 0.01, ***p < 0.001, ****p < 0.0001, ns indicates no statistically significant difference.

**Data S3.** Protein expression results of ERK and Wnt pathway after GNB2 knockdown and statistical analysis of Western blot results. (A, B) Protein expression results show the knockdown effect of GNB2 in CRC cells. (C, D) Protein expression levels of pERK and ERK after GNB2 knockdown. (E, F) Protein expression levels of APC, β‐catenin, and pβ‐catenin after GNB2 knockdown. (G) Figure 8B Western blot statistical analysis results. (H) Figure 8F Western blot statistical analysis results. (I) Figure 8H Western blot statistical analysis results. (J) Figure 8J Western blot statistical analysis results, *p < 0.05, **p < 0.01, ***p < 0.001, ****p < 0.0001, ns indicates no statistically significant difference.

**Data S4.** Graphical abstract.

## Data Availability

All relevant data are within the manuscript and its Additional files. The data are available from the corresponding author on reasonable request.

## References

[1] Siegel RL , Wagle NS , Cercek A , Smith RA , Jemal A . Colorectal cancer statistics, 2023. CA Cancer J Clin. 2023;3:233‐254.10.3322/caac.2177236856579

[2] Kiran NS , Yashaswini C , Maheshwari R , Bhattacharya S , Prajapati BG . Advances in precision medicine approaches for colorectal cancer: from molecular profiling to targeted therapies. ACS Pharmacol Transl Sci. 2024;7(4):967‐990.38633600 10.1021/acsptsci.4c00008PMC11019743

[3] Zhu Y , Zhou B , Hu X , et al. LncRNA LINC00942 promotes chemoresistance in gastric cancer by suppressing MSI2 degradation to enhance c‐Myc mRNA stability. Clin Transl Med. 2022;1:e703.10.1002/ctm2.703PMC878598435073459

[4] Yao ZT , Yang YM , Sun MM , et al. New insights into the interplay between long non‐coding RNAs and RNA‐binding proteins in cancer. Cancer Commun (Lond). 2022;2:117‐140.10.1002/cac2.12254PMC882259435019235

RETRACTED

[5] Hashemi M , Moosavi MS , Abed HM , et al. Long non‐coding RNA (lncRNA) H19 in human cancer: from proliferation and metastasis to therapy. Pharmacol Res. 2022;184:106418.36038043 10.1016/j.phrs.2022.106418

[6] Akhbari MH , Zafari Z , Sheykhhasan M . Competing endogenous RNAs (ceRNAs) in colorectal cancer: a review. Expert Rev Mol Med. 2022;24:e27.35748050 10.1017/erm.2022.21

[7] Zhang X , Ma D , Xuan B , et al. LncRNA CACClnc promotes chemoresistance of colorectal cancer by modulating alternative splicing of RAD51. Oncogene. 2023;17:1374‐1391.10.1038/s41388-023-02657-y36906654

[8] Zhou L , Jiang J , Huang Z , et al. Hypoxia‐induced lncRNA STEAP3‐AS1 activates Wnt/beta‐catenin signaling to promote colorectal cancer progression by preventing m(6)A‐mediated degradation of STEAP3 mRNA. Mol Cancer. 2022;1:168.10.1186/s12943-022-01638-1PMC939228735986274

[9] Wu QN , Luo XJ , Liu J , et al. MYC‐activated LncRNA MNX1‐AS1 promotes the progression of colorectal cancer by stabilizing YB1. Cancer Res. 2021;10:2636‐2650.10.1158/0008-5472.CAN-20-374733782099

[10] Mahdi Khanifar M , Zafari Z , Sheykhhasan M . Crosstalk between long non‐coding RNAs and p53 signaling pathway in colorectal cancer: a review study. Pathol Res Pract. 2023;249:154756.37611430 10.1016/j.prp.2023.154756

[11] Zhang J , Jiang Y , Zhu J , et al. Overexpression of long non‐coding RNA colon cancer‐associated transcript 2 is associated with advanced tumor progression and poor prognosis in patients with colorectal cancer. Oncol Lett. 2017;6:6907‐6914.10.3892/ol.2017.7049PMC569671729181105

[12] Galamb O , Bartak BK , Kalmar A , Nagy ZB , Szigeti KA , et al. Diagnostic and prognostic potential of tissue and circulating long non‐coding RNAs in colorectal tumors. World J Gastroenterol. 2019;34:5026‐5048.10.3748/wjg.v25.i34.5026PMC674728631558855

[13] Shi Y , Wang J , Tao S , et al. Yang. miR‐142‐3p improves paclitaxel sensitivity in resistant breast cancer by inhibiting autophagy through the GNB2‐AKT‐mTOR pathway. Cell Signal. 2023;103:110566.36539001 10.1016/j.cellsig.2022.110566

[14] Yoda A , Adelmant G , Tamburini J , et al. Mutations in G protein beta subunits promote transformation and kinase inhibitor resistance. Nat Med. 2015;1:71‐75.10.1038/nm.3751PMC428911525485910

[15] Chen S , Wu H , Lv N , et al. LncRNA CCAT2 predicts poor prognosis and regulates growth and metastasis in small‐cell lung cancer. Biomed Pharmacother. 2016;82:583‐588.27470400 10.1016/j.biopha.2016.05.017

[16] Zhao Z , Wang J , Wang S , Chang H , Zhang T , Qu J . LncRNA CCAT2 promotes tumorigenesis by over‐expressed Pokemon in non‐small cell lung cancer. Biomed Pharmacother. 2017;87:692‐697.28088736 10.1016/j.biopha.2016.12.122

RETRACTED

[17] Huang S , Qing C , Huang Z , Zhu Y . The long non‐coding RNA CCAT2 is up‐regulated in ovarian cancer and associated with poor prognosis. Diagn Pathol. 2016;1:49.10.1186/s13000-016-0499-xPMC490139727283598

[18] Deng H , Gao J , Cao B , et al. LncRNA CCAT2 promotes malignant progression of metastatic gastric cancer through regulating CD44 alternative splicing. Cell Oncol (Dordr). 2023;6:1675‐1690.10.1007/s13402-023-00835-4PMC1297463037354353

[19] Chen M , Zhao M , Hou Y , Zhu B . Expression of lncRNA CCAT2 in children with neuroblastoma and its effect on cancer cell growth. Mol Cell Biochem. 2021;4:1871‐1879.10.1007/s11010-020-04042-933475889

[20] He P , Xiong G , Guo W , Jiang G , Li Y , Li H . Long non‐coding RNA CCAT2 promotes prostate cancer cell proliferation and invasion by regulating the Wnt/beta‐catenin signaling pathway. Oncol Lett. 2020;4:97.10.3892/ol.2020.11958PMC743912832831916

[21] Moradi F , Mohajerani F , Sadeghizadeh M . CCAT2 knockdown inhibits cell growth, and migration and promotes apoptosis through regulating the hsa‐mir‐145‐5p/AKT3/mTOR axis in tamoxifen‐resistant MCF7 cells. Life Sci. 2022;311:121183.36375570 10.1016/j.lfs.2022.121183

[22] Chen B , Dragomir MP , Fabris L , et al. The long noncoding RNA CCAT2 induces chromosomal instability through BOP1‐AURKB signaling. Gastroenterology. 2020;159(6):2146‐2162. e33.32805281 10.1053/j.gastro.2020.08.018PMC7725986

[23] Zhao H , Ming T , Tang S , et al. Wnt signaling in colorectal cancer: pathogenic role and therapeutic target. Mol Cancer. 2022;1:144.10.1186/s12943-022-01616-7PMC928113235836256

[24] Yu QY , Han Y , Lu JH , Sun YJ , Liao XH . Liao.NRP1 regulates autophagy and proliferation of gastric cancer through Wnt/beta‐catenin signaling pathway. Aging. 2023;17:8613‐8629.10.18632/aging.204560PMC1052236437702613

[25] Zhou Y , Xu J , Luo H , Meng X , Chen M , Zhu D . Wnt signaling pathway in cancer immunotherapy. Cancer Lett. 2022;525:84‐96.34740608 10.1016/j.canlet.2021.10.034

[26] Hemmati‐Dinarvand M , Ahmadvand H , Seghatoleslam A . Nitazoxanide and cancer drug resistance: targeting Wnt/beta‐catenin signaling pathway. Arch Med Res. 2022;3:263‐270.10.1016/j.arcmed.2021.12.00134937659

[27] Chen Y , Chen M , Deng K . Blocking the Wnt/beta‐catenin signaling pathway to treat colorectal cancer: strategies to improve current therapies (review). Int J Oncol. 2023;62(2):24.36579676 10.3892/ijo.2022.5472PMC9854240

[28] Zhu Y , Li X . Advances of Wnt Signalling pathway in colorectal cancer. Cells. 2023;12(3):447.36766788 10.3390/cells12030447PMC9913588

[29] Zhu J , Cao K , Zhang P . J Ma.LINC00669 promotes lung adenocarcinoma growth by stimulating the Wnt/β‐catenin signaling pathway. Cancer Med. 2023;12(7):9005‐9023.36621836 10.1002/cam4.5604PMC10134358

RETRACTED

[30] Zhang K , Liu P , Tang H , et al. AFAP1‐AS1 promotes epithelial‐mesenchymal transition and tumorigenesis through Wnt/β‐catenin signaling pathway in triple‐negative breast cancer. Front Pharmacol. 2018;9:1248.30505272 10.3389/fphar.2018.01248PMC6250734

[31] Tang Y , Tian W , Zheng S , et al. Dissection of FOXO1‐induced LYPLAL1‐DT impeding triple‐negative breast cancer progression via mediating hnRNPK/β‐catenin complex. Research (Wash DC). 2023;6:289.10.34133/research.0289PMC1072629338111678

[32] Chen S , Ji L , Wang Y , et al. lncRNA RMST suppresses the progression of colorectal cancer by competitively binding to the miR‐27a‐3p/RXRα axis and inactivating the Wnt signaling pathway. Acta Biochim Biophys Sin Shanghai. 2023;55(5):726‐735.37246895 10.3724/abbs.2023065PMC10281887

[33] Zhou L , Jiang J , Huang Z , et al. Hypoxia‐induced lncRNA STEAP3‐AS1 activates Wnt/β‐catenin signaling to promote colorectal cancer progression by preventing m6A‐mediated degradation of STEAP3 mRNA. Mol Cancer. 2022;21(1):168.35986274 10.1186/s12943-022-01638-1PMC9392287

[34] Fey D , Matallanas D , Rauch J , Rukhlenko OS , Kholodenko BN . The complexities and versatility of the RAS‐to‐ERK signaling system in normal and cancer cells. Semin Cell Dev Biol. 2016;58:96‐107.27350026 10.1016/j.semcdb.2016.06.011

[35] Samatar AA , Poulikakos PI . Targeting RAS‐ERK signaling in cancer: promises and challenges. Nat Rev Drug Discov. 2014;12:928‐942.10.1038/nrd428125435214

[36] Guo YJ , Pan WW , Liu SB , Shen ZF , Xu Y , Hu LL . ERK/MAPK signaling pathway and tumorigenesis. Exp Ther Med. 2020;3:1997‐2007.10.3892/etm.2020.8454PMC702716332104259

[37] Zong W , Ju S , Jing R , Cui M . Long non‐coding RNA‐mediated regulation of signaling pathways in gastric cancer. Clin Chem Lab Med. 2018;11:1828‐1837.10.1515/cclm-2017-113929804098

[38] Xie SJ , Diao LT , Cai N , et al. mascRNA and its parent lncRNA MALAT1 promote proliferation and metastasis of hepatocellular carcinoma cells by activating ERK/MAPK signaling pathway. Cell Death Dis. 2021;1:110.10.1038/s41420-021-00497-xPMC812890834001866

[39] Zhang L , Sahar AM , Li C , et al. A detailed multi‐omics analysis of GNB2 gene in human cancers. Braz J Biol. 2022;84:e260169.35730811 10.1590/1519-6984.260169

